# PRISM: A Novel Visual Instrument to Facilitate Self-Reflection and Learning Progress in Undergraduate Dental Education

This article has been retracted.

**DOI:** 10.1155/2022/2009894

**Published:** 2022-08-16

**Authors:** Gerhard Schmalz, Tom Sensky, Henrike Kullmann, Stefan Büchi, Dirk Ziebolz

**Affiliations:** ^1^Department of Cardiology, Endodontology and Periodontology, University of Leipzig, Leipzig, Germany; ^2^Centre for Mental Health, Department of Medicine, Imperial College London, London, UK; ^3^Clinic for Psychotherapy and Psychosomatics “Hohenegg”, Meilen, Switzerland

## Abstract

**Objectives:**

PRISM (Pictorial Representation of Illness and Self-Measure) is a simple visual tool that has been successfully used as a visual metaphor in medicine. In this pilot study, PRISM was used for the first time to test its potential to support self-reflection and expectations of learning in dental students.

**Methods:**

Dental student volunteers (25 3^rd^ year, 10 4^th^ year, and 10 5^th^ year) participated. Using both quantitative and qualitative methods, PRISM interviews were compared with a numerical scale in assessing learning objectives concerning theoretical knowledge, practical skills, interest, and training need in the field of conservative dentistry.

**Results:**

Overall, 71% of total student group stated that they would draw personal consequences for their studies due to participating in the PRISM interviews. Compared to the numeric scales, PRISM was rated as more helpful regarding appraisal of students' theoretical knowledge (*p* = 0.02), practical skills (*p* < 0.01), training needs (*p* < 0.01), importance of dental subspecialties (*p* < 0.01), and facilitating self-reflection (*p* = 0.02). In focus groups, students commented that PRISM fostered the development of a trusting relationship with their teacher. Strengths of PRISM mentioned by the students included being able to observe and manipulate a visual summary of their individual learning needs and seeing their different learning needs in relation to one another.

**Conclusion:**

In this pilot study, dental students evaluated PRISM to be superior against numeric scales. Furthermore, it ameliorated the communication with teachers. The PRISM task is both simple and brief and warrants further exploration as a useful tool for self-reflection in dental education.

## 1. Introduction

A hallmark of all professions is the need to develop theoretical knowledge and practical skills throughout one's career. Such career-long learning is crucially dependent on developing a capacity for effective self-reflection—the professional needs to be able to identify and appraise their learning needs. In dental education, as in the training of other professions, one major aim of teachers is to assist their students to become self-directed healthcare professionals and to initiate a lifelong learning process [1]. Students are seen as self-directed and active partners in their educational environment and should develop trusting relationships with their teachers [2]. This requires continuous self-reflection, what is defined as a process where the students themselves need to get into a critical, exploratory, attentive, and interactive engagement with their own thoughts and activities [3]. Although the influence of self-reflection on academic performance remains controversial, because studies to date have found only a minor effect [4–6], it has been considered to be a core skill in dental education [7].

Four facettes of self-reflection, i.e., habitual action, understanding, reflection, and critical reflection, are explicitly mentioned; these subaspects influence learning approaches, learning goals, and academic performance [8]. The form and content of self-reflection are of practical relevance. Different approaches are available, e.g., self-reflection combined with peer-feedback, video-watching, or expert-feedback [9, 10]. Furthermore, a recent systematic review reported on the available instruments to measure the ability of self-reflection [7]. Thereby, rubrics (or scoring guides), self-reported scales, and observed behavior were differentiated, and it has been concluded that none of these tools can be recommended as single measure [7]. Thus, based on this systematic review and to the authors' knowledge, there is no self-reflection method widely acknowledged as the ‘gold standard.' Therefore, the appropriate approach for self-reflection in dental education still remains a question of theoretical and practical interest.

The present study is a ‘proof of concept' investigation to determine whether a novel measure warrants further investigation as a tool to facilitate self-reflection. PRISM (Pictorial Representation of Illness and Self-Measure) is a visual instrument that has been developed in the field of medicine to assess patients' appraisal of their suffering due to illness [11] and to facilitate discussion between patient and clinician about the patient's experience of illness [12]. More recently, PRISM has been applied more widely, including in coaching. Thereby coaching and self-reflection are closely related to each other; on the one hand, coaching facilitates self-reflection [13] and on the other hand, self-assessment and developing reflective skills is a part of the coaching process [14]. Growing experience in its use indicates that PRISM functions as a visual metaphor and it is this property, which allows it to generate personally salient information [15]. Several applications beside of the original task are the usage of PRISM in context of alcohol abuse [16], acceptance of vaccinations and perceived risk of travel-related risks [17], or perceived work stress of anesthesiologists [18]. Accordingly, PRISM has the potential to be used in new fields of research and could be relevant for other contexts, including student self-evaluation of learning progress.

Up to the knowledge of the authors, there have been no publications to date describing any application of PRISM in education. The present study is aimed at assessing PRISM as a tool to facilitate self-reflection in undergraduate dental education. Both quantitative and qualitative data were collected to evaluate the strengths and limitations of the application of PRISM. It was hypothesized that PRISM would be appraised by students as a helpful tool for self-reflection. It was also anticipated that PRISM might have a positive effect on student-teacher communications.

## 2. Methods

### 2.1. Study Design

The study was cross-sectional pilot study, using both qualitative and quantitative methods and involving three groups of dental students at different stages of their training. The study protocol was reviewed and approved by the ethics committee of the medical faculty of University of Leipzig, Germany (No.: 117/20-ek). All participants were informed verbally and in writing about the study and provided their written informed consent for participation. The general study flow is shown in Figure 1.

### 2.2. Participants and Groups

All students who participated in the study were volunteers, and all were in the clinical years of their dental studies. Twenty-five 3^rd^ year students were included from a group, which had completed a clinical simulation course in conservative dentistry. Ten students were included from each of the 4^th^ and 5^th^ years, at the end of their clinical courses in conservative dentistry and periodontology, respectively. Students resetting these courses were not permitted to participate—all participants were doing their respective courses for the first time. The study was performed between June and September 2020. To ensure safety against the background of the COVID-19 pandemic, the interviewer and student were separated by a Plexiglas pane and wore medical gloves and all instruments were disinfected at each exchange.

### 2.3. The PRISM Task

Initially, PRISM originates from the field of psychology/psychosomatic medicine [11, 12]. PRISM is a visual metaphor of the relationship between a subject and associated objects in a defined context [15]. A white metal board (210 × 297 mm) represents the Context, in this case “Your dental studies.” A fixed yellow circle (7 cm in diameter) in the bottom right hand corner of the board, represents the Subject (“myself as a X-year dental student”). Magnetic disks, 5 cm in diameter and in different colors, represent the Objects—different aspects of dental studies like “your practical skills in periodontology” or “your theoretical knowledge of conservative dentistry” (see Figure 2). Participants are simply instructed to place each Object disk on the board to reflect their appraisal of that aspect of their studies. The main quantitative output generated by PRISM is the distance between the Subject and Object. Previous research has indicated that the closer the Object is placed to the Subject, the more salient the participant appraises the Object to be to the Subject in the defined Context [15]. Thus, putting a particular learning objective close “myself as an X-year dental student” means that the student has made good progress with that objective and regards it as a successful part of her/his learning. The crucial difference between PRISM and other quantitative measures is that its visual format coupled with the simple instructions mean that where the Object disks are placed on the board is inevitably personally salient to the individual participant. Examples of completed PRISM tasks are shown in Figures 3 and 4.

### 2.4. PRISM Interviews

The PRISM interviews were additional to the students' scheduled learning. Generally, all students underwent practical courses in conservative dentistry, including the treatment of patients or its simulation, respectively. These courses are regularly evaluated by questionnaires with numeric scales at the end of the term. Both, PRISM and the self-reflection questionnaire, in the current study were used in addition to the regular curriculum. All PRISM interviews were performed in the same setting by a dentist trained in the use of PRISM, who was not directly involved in the routine appraisal included in the respective course. All participants had three PRISM interviews within one week, each lasting 10-12 minutes, with exactly the same tasks in each interview. Three interviews were included to assess the reproducibility of PRISM (the PRISM data will be reported separately). Moreover, multiple interviews were applied to give students the opportunity to get more experienced and accustomed with the method. At the first interview, the PRISM task was explained to all participating students and one example question given (“The white board represents your life and the yellow fixed circle represents you. Imagine this blue disk is burger and this green disc is broccoli. Where would you put these disks to reflect how much do you like it at the moment?”). At the subsequent interviews, the PRISM task was again explained briefly. In each interview, the students were asked to place 1-5 object disks including 16 different questions on the PRISM board reflecting their theoretical knowledge, practical skills, interests, and training needs and perception of different fields in conservative dentistry. Each student was asked the same 16 questions. The topics of those questions were chosen according to validated evaluation questionnaires, which are used during the dental curriculum to evaluate the clinical courses. All potential questions were screened and discussed in the author group and finally used for the interviews. A separate validation step for the task was not performed. For example, “How do you rate your practical skills in the field of periodontology?,” “How do you rate your interest in the field of endodontology?,” or “How much training do you think to need in the field of cariology?” were used as questions for the PRISM task. The nearer the object was placed to the subject, the better students appraised their practical skills or the greater their interest. With the “training need” questions, the further these Object disks were from “Myself as a X-year dental student,” the greater the appraised training need (a separate and specific instruction was given to the students about this). Ten of the 3^rd^ year students and all the 4^th^ year student participants had an additional PRISM interview six weeks after the third interview, which was videotaped. For this, 5^th^ year students could not be included as they were in their final exams at that time. This interview was reduced to five different questions, covering theoretical knowledge, practical skills, interest, training needs, and importance of each of the five subspecialties of conservative dentistry (cariology, periodontology, endodontology, restorative dentistry, and prevention). This fourth interview included a discussion with each student about why they had placed their disks where they had on the PRISM board and how these placements might be interpreted in terms of the student's self-appraisal of successful learning and of learning needs.

### 2.5. Control Self-Reflection Measure

As a control, the same questions about appraisal asked using PRISM were asked on a 0-10 numerical scale after the fourth PRISM interview. The students were already accustomed to using numerical scales for evaluation, as scales are used during the dental curriculum after each student course for evaluation. These evaluation tasks for the clinical courses were the basis to develop the topics of interest in the current study. The questionnaire was composed in full accordance to the PRISM task and included exactly the same wording of questions, which were answered on the numeric scale. No separate validation step was performed.

### 2.6. Scales to Evaluate Use of PRISM

After the third PRISM interview, all participants were asked to rate on a scale between 0 (very low) and 10 (very high) the extent, to which they considered that the PRISM task had been helpful in their appraisal of their own competencies, including theoretical knowledge, practical skills, interest, and training needs. In other words, students rated the extent, to which PRISM had helped them better appraise their competencies. For the 20 students who had the videotaped PRISM interview, they were all asked immediately after the PRISM interview to rate the same questions about appraisal as used in the PRISM interview on a 0-10 scale as control (see above). Afterwards, students rated on a scale between 0 (very low) and 10 (very high), to what extent they perceived an impact of PRISM and/or the numerical scales on their perception of own competencies.

### 2.7. Focus Group Discussion

To gain further insights into the students' perspective, two focus groups were held. Only the 20 students, who had participated in all four PRISM interviews were invited, and eight students from each of the two year groups agreed to participate. Two investigators watched the PRISM interview videotapes and the topics for group discussion were generated from these. These topics were as follows: the relationship between student and teacher and whether this is influenced by the PRISM method; the relative importance for a successful interview of the three elements—PRISM method, interviewer, and setting; whether the relationship with the interviewer built up in the PRISM interview was seen as personal or as topic-related (i.e., course-specific content explored in the PRISM task); strengths and limitations of PRISM method. First, each topic was introduced in the focus groups and examples from the video analysis were explained. Afterwards, the groups discussed each topic individually. Based on this discussion, the groups had the task to formulate main statements regarding the respective topic. These resulting summary statements or conclusions were formulated within the focus group to reflect the group consensus and to include each participant actively in the process of evaluating the method. Each summary statement has been finally rated by the whole focus group and was only fixed if all eight participants agreed, and otherwise, it was modified until a full consensus was achieved. Thus, only consensus statements, which were confirmed by all of the focus group participants, were finally formulated.

### 2.8. Statistical Analysis

The statistical analysis has been performed with SPSS for Windows, version 24.0 (SPSS Inc., U.S.A.). Values are presented as mean values with standard deviation or percentage, respectively. Normal distribution was tested with the Shapiro-Wilk test. Thereby, the four questions regarding competencies (theoretical knowledge, practical skills, interest, and training needs) were normal distributed (p>0.05), while the rest showed nonnormal distribution. Based on normal distribution, Wilcoxon-test or *t*-test was applied. The significance level was set at *p* < 0.05.

## 3. Results

### 3.1. Participants

In total, 45 students were included, with a mean age of 23.2 ± 3.1 years (40% male gender). Of these participants, 25 students in 3^rd^ year (age 22.9 ± 2.9 years, 32% male), as well as 10 students in 4^th^ (age 23.5 ± 2.9 years, 50% male) and 5^th^ year (age 24.9 ± 2.8 years, 50% male) took part in the study. Based on the total numbers of the respective study years, 48% (25/52) of 3^rd^ year, 22% (10/46) of 4^th^ year, and 23% (10/44) of 5^th^ year students participated in this study.

### 3.2. Evaluation of PRISM after 3 Interviews

The results of the evaluation of PRISM in the total group are shown in Table 1. Overall, 71% of total group stated that they would draw personal consequences from the PRISM interviews for their further study in dentistry. The distribution of ratings (0-4, 5, or 6-10) showed more than half of the students rated PRISM as positive (value 6-10) for all questions asked. No significant gender differences were found (Table S1).

### 3.3. Comparison between PRISM and Numeric Scale

PRISM was rated to be significantly more helpful than the numerical scale for the perception of students' self-reflection competencies (Table 2). Significantly, more students said that they would draw personal consequences for their learning from PRISM than from the numerical scales (80% vs. 50%, *p* < 0.01). Moreover, PRISM was rated to be a better tool for self-reflection than the numeric scale (Table 2).

### 3.4. Focus Group Discussion

A summary of focus group results is given in Table 3. The relationship between the student and teacher was stated as important, and PRISM was rated as supporting the building of this relationship. In evaluating the success of the interview, the students gave similar weights to the PRISM method and to the interviewer. However, the interviewer placed more importance on the PRISM method. Major strengths for the students were being able to scale their appraisals individually and to gain a visual summary of their appraisals, including being able to gain a picture of different topics in relation to one another (Table 3). The need for explanation to understand the PRISM task was identified as a limitation of PRISM. The interviewer perceived a high benefit, especially due to supported relationship building and the fact that PRISM was useful to gain a deeper understanding of the students' perspective.

## 4. Discussion

PRISM was originally developed to better understand the illness experience of individual patients. However, perhaps encouraged by its novelty as a visual metaphor, an increasingly wide range of applications has been reported and it has been proposed as potentially useful in coaching [15]. This led to the present study, the first reported application of this type for PRISM.

This study had modest aims, to assess the acceptability and potential utility of PRISM as a tool for appraisal in undergraduate dental education. The small sample was in keeping with the aims of the study as a preliminary investigation. However, the fact that the student participants were all volunteers could have biased their responses. Moreover, the participants were only a minority of the respective cohort and thus its representativeness is limited. Again in keeping with the modest aims of the study, no attempt was made to integrate the PRISM task into the students' teaching programme or curriculum—this would have been premature before gathering basic data on potential acceptability and utility. The fact that the PRISM task was repeated three or four times (to gather data in the reproducibility of its results, to be reported separately as part of the PRISM outputs) could also have influenced students' responses. The study was performed during the COVID-19 pandemic, whereby specific measures to prevent infections had to be applied. This might also limit the generalizability of the findings. A further limitation, which could not be avoided in the study design, was asking the students to use and assess the control appraisal tool (the numerical scale) after they had gained experience of PRISM—this could have biased their responses. It is known that the original PRISM task has a good test-retest reliability and interrater reliability [11, 19]. Furthermore, the PRISM method is sensitive for change over time [15]. This would be also of interest in context of education and will be addressed in a subsequent project. Generally, the PRISM task is originally understood by the vast majority of patients [11]; the questions in the current study were sometimes quite complex and therefore more challenging. Several other methodical limitations require consideration. Students were only asked, whether they would draw consequences from the PRISM task, but not which consequences would that be. Furthermore, it is difficult to state what is a “positive” result at a scale between 0 and 10 by focusing on the mean values. For this rationale, the distribution of ratings lower and higher than 5 was presented as well, whereby results of 6-10 might be considered as merit or benefit, respectively. Although the topics included in the PRISM task and self-reflection questionnaire were chosen in accordance to available and common evaluation procedures, no validation of the measures was performed. The qualitative data in the current study were presented as consensus statements, which were formulated by the participants. The topics for these statements were chosen based on video analysis of the interviews, but a validation was not performed. The authors decided to use this consensus form to allow statements reflecting the students' perspective on PRISM as a tool for dental education for the first time. Overall, this limits the usage of the applied instruments and the generalizability of the findings. Future studies should use more valid qualitative analysis methods, as the applied methodology cannot be referenced and is therefore somewhat biased.

Allowing for these limitations, the current study's results, both quantitative (Table 1) and qualitative (Table 3) indicate that the students engaged well with PRISM task and found it helpful in appraising their competencies, and superior to a numerical scale (Table 2).

The majority of the students rated PRISM as helpful in appraising their competencies and 71% endorsed that they had learned from the PRISM task something relevant to their further studies (Table 1). The students appreciated PRISM as a visual tool and one, which is ‘calibrated' by each individual student, in terms of where the Object disks are placed. As a visual metaphor, the placement of each Object disk depends crucially on the individual's reflections about that Object. While it is possible to endorse a number on a 0-10 scale without giving the task much thought, this is not possible for PRISM, and this was reflected in the students' responses. Both 3^rd^ and 4^th^ year students considered that the PRISM task and the interviewer were important, although the 4^th^ year students gave more weight to the setting of the task. Students in 4^th^ year had more experience of appraisals in their dental studies, while for the 3^rd^ year students, this was their first experience of appraisal. The context of the PRISM task was therefore not new for the 4^th^ year students; hence, they may have been more discriminating than their 3^rd^ year colleagues. Overall, the strengths of PRISM identified by the students (Table 3) are consistent with those previously reported [15]. Thereby, the main benefit was seen in its individuality and the benefit of the concept of a metaphor. A visual metaphor allows increased flexibility in thinking and interpretation, what encourages creative thinking [20]. It has already been described that participants using such a visual metaphor are able to construct and appraise external representations of their own perspective and knowledge [21]. Additionally, the usage of this visual metaphor enables informants thinking differently, leading to different conclusions [22]. This underlines the individuality of the PRISM task. The visual methaphorization is thereby a very special approach. Metaphors, which are visualized in this way, cannot be easily and blanked interpreted, but a specific understanding of the metaphor is needed [15]. Thereby, such a visual metaphor can only be understood in a personal context [23]. While a rubric tool, especially numeric scales are quite general and primarily focused on objectivating an evaluation for the teacher, PRISM interviews were on a personally salient way, in which the student experienced that his interests and view are relevant for the teacher.

Both the students and the interviewer noted the potential of PRISM to support the relationship between student and teacher. One of the earliest observations in using PRISM was its positive effect on communications between patients and clinicians [12]. In the present context, having the completed PRISM task as a visual summary of competencies is likely to facilitate discussion between student and teacher. Having needed to reflect on where to place each Object disk, the student can give a succinct answer to the question ‘Why did you put the [Object] disk there?.' Including multiple Object disks can extend the discussion, for example to agreeing priorities.

The PRISM task is very simple, as illustrated by the Figures 2 and 3. In the past, changes have been introduced to PRISM, which make it more complicated, for example giving participants a choice of differently sized Object disks. Such changes have altered the outcome of the task [15]. This highlights the importance for PRISM, as for any other metaphor, of giving the participant the minimum information required to make a personally salient interpretation of the metaphor, but no extraneous information [23, 24]. It is crucial at the start of the task for the participant and interviewer to have a shared, explicit, and clear understanding about what are the Subject, Object, and Context of the task. In the authors' experience, it is often necessary to pilot the task to check this. For example, in the present study, defining the Subject as ‘myself as a dental student' is not as precise as ‘myself as an X-year dental student,' and these may yield different responses. As PRISM requires more skills and time than conventional numeric scales, potentially limiting the ability of PRISM to be promoted among students with heavy learning tasks and very little free time. On the one hand, PRISM interviews were associated with a time effort between 10 and 12 minutes, what appears an efficient time span for relationship building and reflection with the teacher. On the other hand, a software based application of PRISM is available, although this cannot include the “haptic” experience of placing an object disk. Therefore, this could be an interesting practical approach to include PRISM in education, which would require subsequent evaluation.

As already mentioned, this is the first application of PRISM method in education. Accordingly, comparable studies are not available, yet. The current study was performed in a cohort of dental students from three different years of study. In tendency, students in the earlier years of studies (3^rd^ and 4^th^ year, Table 1) experienced a higher benefit from PRISM. This is in line with the literature, showing that reflective thinking can be fostered especially in younger students [25]. Self-reflection in the early years of dental study was reported to increase the awareness and premises the context of learning environment of the students [25]. Although, statistical testing between the three groups (3^rd^, 4^th^, and 5^th^ year) was omitted in the current study, due to limited sample size, it might be recommendable to apply PRISM interviews in the early dental study terms.

PRISM was found to be superior against numeric scale regarding self-reflection in the current pilot study. A numeric scale (or scoring) as rubric tool for self-reflection has been evaluated in several studies [7]. A systematic review did not confirm a superiority of any instrument [7]. Different other forms or strategies of self-reflection are available. Continuous self-reflection via logbook, to help students learning from their own experiences, was found to increase student's knowledge and skills [26]. Furthermore, peer-feedback combined with self-reflection was able to increase students' performance [10]. Similarly, watching a video tape of their own patient communication was experienced to be helpful for self-reflection for dental students, which is an approach of self-observed behaviour [9]. This approach of students watching their own video implies a visualization, which can be linked to PRISM, whereby the own perspective is reflected using a visual metaphor. With regard to the different facettes of reflection [8], PRISM appears to support critical reflection of the own view. This is especially supported by the focus group finding that students reported that they needed to “position myself to my own individual perception” for the first time in their dental education.

An important study concluded that the assessment of student's perspective is of high relevance for dental education, making research projects needed, which assess this perspective by the respective feedback and perceptions of the students [27]. This approach is picked up in the PRISM method and extended on visualization of the student's perspective for the student himself. This visualization was positively emphasized in the focus group discussions and seems to be a major strength of PRISM method in dental education. Moreover, one strength of PRISM was that fostered relationship building between teacher and student and supported respectful relationship at eye level; this fulfilled the demand of Radford et al., stating that students gain from a learning environment, in which they perceive to be an essential and respected part [2]. Besides this, the interpretation of PRISM findings was experienced to be very individual. Although this can be seen as a challenge for the teacher (and possibly the student himself) to understand the students view, this can also be a chance for changing some concepts of dental education. In the few last years, individualized education has been discussed as a promising approach [28, 29]. By assessing the students' perspective by means of PRISM, training needs, and interests of the students can be helpful to individualize the teaching offers. Furthermore, the motivation of students in medical education is an issue of practical interest and strategies to positively influence students' motivation are reported [30]. Especially assessing the individual interests and training needs by the student himself during PRISM interviews might be helpful to foster intrinsic motivation for learning in dental study. Thereby, PRISM can be seen as a tool, which helps the teacher to support or assist the student in his own process of personal advancement during study. Accordingly, it is less a teaching, but more a coaching tool, what appears a contemporary approach in education [31]. As stated in the introduction, self-reflection is mandatory for the coaching process, alongside with relationship building [13, 14], which is also supported by the PRISM task.

## 5. Conclusion

Undergraduate dental students perceived the use of PRISM was helpful for self-reflection and superior against a numeric scale, and the visual metaphor of students own perspective was a major strength. Within the limitations, the results of this pilot study are sufficiently encouraging to warrant further investigation of PRISM as a potentially useful tool for self-reflection and appraisal in dental education.

## Figures and Tables

**Figure 1:** Study flow of interviews and evaluation steps with the respective students.

**Figure 2:** Principle of PRISM. The PRISM plate is the Context. The yellow Subject disc is a fixed point on the plate. The student is asked to place one or more Object disks on the plate (for example, ‘my practical skills in ….”). The distance between Subject and Object yields a quantitative measure, and can be used for self-reflection and in discussions between student and appraiser.

**Figure 3:** Examples of PRISM interview responses. (a) The results of a student for “how do you appraise your practical skills in the whole field of conservative dentistry (grey).” (b) The result of the same student for subspecialties of conservative dentistry: “how do you appraise your practical skills in periodontology (yellow), cariology and restorative dentistry (blue), endodontology (violet) and preventive dentistry (green).” Note that PRISM allows the differentiation of the subspecialties as well as giving a ‘summary' measure. (c) The results of another student for “how do you appraise your practical (grey) and theoretical (black) skills in the field of conservative dentistry?.” (d) The results of the same student for “how do you appraise your remaining training needs in conservative dentistry (red; the greater the distance from the Subject circle, the greater the appraised training need). While the skills and knowledge are appraised as good (c), the training need is still high (d).

**Figure 4:** The individuality in answering the PRISM task is a major strength. (a) A stack of several object discs, which have nearly the same perceived importance for the student. (b) The possibility of place one disc (blue) in the center, leading to the placement of the further object disc in relation to the subject disc, but also in relation to this subject disc. (c) Another pattern of Object disks.

**Table 1:** Results of the evaluation of PRISM for the total sample. Values are rated between 0: very low and 10: very high.

	Total sample (*n* = 45)	Rated values		
		0-4	5	6-10
*The assessment with PRISM 0-10 was helpful for my appraisal of…*				
My theoretical knowledge	5.9 ± 2.4	22% (10)	22% (10)	56% (25)
My practical skills	5.8 ± 2.8	24% (11)	18% (8)	58% (26)
My interest	6.1 ± 2.6	24% (11)	4% (2)	71% (32)
My training needs	5.9 ± 2.5	27% (12)	13% (6)	60% (27)
Personal consequences for further study (yes/no)	71%	—		

**Table 2:** Comparison of the self-perceived helpfulness of PRISM and a numeric scale (0-10) in the participants of 3^rd^ and 4^th^ year, who underwent the video-taped PRISM interview (*n* = 20).

Topic	PRISM		Numeric scale 0-10		*p* value
	Mean value	Rating 6-10	Mean value	Rating 6-10	
*The assessment with PRISM/numeric scale 0-10 was helpful for the appraisal of…*					
My theoretical knowledge	6.8 ± 1.9	80% (16)	5.2 ± 2.2	45% (9)	**0.02** ^**a**^^∗^
My practical skills	6.6 ± 1.7	70% (14)	5.1 ± 2.7	45% (9)	**<0.01** ^∗^
My interest	6.9 ± 2.3	70% (14)	4.5 ± 2.5	30% (6)	0.12^∗^
My training needs	7.3 ± 2.1	85% (17)	5.6 ± 2.7	45% (9)	**<0.01** ^∗^
Importance of subareas of dentistry	6.4 ± 2.7	70% (14)	4.7 ± 2.4	35% (7)	**<0.01** ^∗∗^
Personal consequences for further study (yes/no)	80%	—	50%	—	**<0.01** ^∗∗^
Is a good tool for self-reflection	8.5 ± 1.3	100% (20)	5.6 ± 2.5	50% (10)	**0.02** ^∗∗^

^a^The statistics refer to the differences between means. ^∗^*t*-test. ^∗∗^Wilcoxon test.

**Table 3:** Results (consensus statements) of the focus group discussions plus interviewer's comments. The points listed in the tables reflect the consensus statements of the whole focus group.

Topic	Group I interviews in 3rd year (*n* = 8)	Group II interviews in 4th year (*n* = 8)	Interviewer's experiences
Relationship teacher–student and how PRISM can affect this	(i) Very important for success during study (ii) “If you like your teacher, you like to listen to your teacher” (iii) Personal contact of importance for relationship (iv) PRISM can serve as an appropriate basis for relationship (v) PRISM makes relationship building easier	(i) Relationship has more influence on learning than the content (ii) Respectful relationship brings perception of safety and avoids fear, in contrast fear leads to averting the field (iii) PRISM brings a personal shared level and the feeling that student's view is valued (iv) PRISM supports relationship building	(i) Very important for bond of trust in the clinical courses of dental study (ii) PRISM opened the contact and served as a good basis for forming relationship with students (iii) Students trended to open up easily by transferring the level of communication on PRISM (iv) PRISM makes relationship building easier (v) Students were not only able to summarize their learning needs but also to view them as an observer
Importance of PRISM method, interviewer, and setting for successful interview	(i) Depends on the interviewer (ii) Setting of minor relevance (iii) 49% PRISM, 49% interviewer, 2% setting	(i) Setting is important to create openness and makes relationship to interviewer easier (or more difficult) (ii) 42.5% PRISM, 42.5% interviewer, 15% setting	(i) Most importance is by PRISM method, because it facilitates the interview (ii) 65% PRISM, 30% interviewer, 5% setting
Personal or issue-related relationship due PRISM interview	(i) Both, personal and factual equally, the more PRISM interviews, the more a personal relationship is built	(i) Primarily factual because of the thematic background, the more PRISM interviews, the greater a sense of security and personal relationship	(i) More personal relationship than factual (ii) The more interviews, the more personal the relationship
Strengths of PRISM method	(i) Being able to observe and manipulate a visual summary of learning needs (ii) Individual scales for different questions (iii) Visual and haptic (iv) Individual interpretation (v) Helpful for self-evaluation and self–reflection (vi) More useful than numerical or percentage scales (vii) Visualizing the relationship between different objects (viii) Visualizing a development process for yourself	(i) Being able to observe and manipulate a visual summary of learning needs visualization of an intuitive placement of the object disk allows an individual perspective (ii) Self-reflection and direct visualization of the learning topic (iii) Individual and also nuanced (iv) Personally salient appraisal (v) Preferred to evaluation based on numerical scales	(i) Being able to observe and manipulate a visual summary of learning needs freedom to reflect student's own view on an topic, unbound by numerical values (ii) Helps the teacher to gain more understanding from the students´ perspective (iii) Haptic and visual method and use of metaphor facilitate self-reflection and –evaluation process by students and teacher
Limitations of PRISM	(i) Needs more explanation to understand the method compared to a numeric scale	(i) Needs explanation and training to understand the method (ii) More time consuming than evaluation using numeric scale	(i) Responses individual and can therefore be difficult to interpret (ii) Vulnerable to subtle influences e.g. precise wording of PRISM introduction and task (iii) More time consuming than using a numeric scale

## Data Availability

The datasets used and/or analyzed during the current study are available from the corresponding author on reasonable request. The data are not publically available, because of the psedonymization and data protection guidelines according to the ethics approval.

## Supplementary Materials

Supplementary Materials Table S1: gender depending differences in the total cohort in results of the evaluation of PRISM for the total cohort. Values are rated between 0: very low and 10: very high.
